# Association of Incidence between Pancreatic Adipose Infiltration and Metabolic Syndrome: A Literature Review and Meta-analysis

**DOI:** 10.1155/2021/5747558

**Published:** 2021-11-05

**Authors:** Ying Zhang, Jing Li, Youqing Xu

**Affiliations:** Department of Gastroenterology, Beijing Tiantan Hospital, Capital Medical University, Fengtai District, Beijing 100070, China

## Abstract

**Objective:**

To investigate association of incidence between pancreatic adipose infiltration and metabolic syndrome (METS).

**Methods:**

We searched PubMed, Embase, Cochrane Library, and Web of Science databases up to July 2021. We compared incidence rate of METS between adults with and without pancreatic adipose infiltration, along with their clinical features, such as fasting blood glucose (FBG), triglyceride (TG), high-density lipoprotein (HDL), and hypertension (HTN). Cross-sectional study, cohort study, and case control study were included. Two investigators independently completed study selection, data extraction, and risk of bias assessment.

**Results:**

Eleven eligible studies that involved 17,127 patients were included, including 8 cross-sectional studies, 2 cohort studies, and 1 case control study. There was a trend of increasing in incidence rate of METS (OR = 2.66, 95% CI: 1.89-3.75) of adults with pancreatic adipose infiltration when compared to those without the disease. There was a trend of increasing in HTN (OR = 1.68, 95% CI: 1.32-2.13) and levels of FBG (SMD = 0.54, 95% CI: 0.35-0.72) and TG (SMD = 0.39, 95% CI: 0.25-0.53) of adults with pancreatic adipose infiltration, while there was a trend of decreasing in HDL level (SMD = −0.29, 95% CI: -0.43~ -0.15).

**Conclusion:**

There was an association of incidence between pancreatic adipose infiltration and METS. Indicators of clinical features related to pancreatic adipose infiltration were more likely to arise, such as FBG and TG levels and HTN, but HDL level tended to decrease.

## 1. Introduction

With higher standards of living, metabolic syndrome (METS) becomes a global health issue attributable to eating high-fat and high-calorie foods and lacking exercise in all age and socioeconomic groups [1, 2]. METS refers to pathological state of metabolic disorder in protein, adipose, and carbohydrate, which is a set of complex disorders containing cardiometabolic syndrome, insulin resistance syndrome, etc. [3, 4]. Obesity, diabetes mellitus (DM), hypertension, dyslipidemia, high blood viscosity, and high uric acid levels may be one of the components of METS.

Ectopic fat can accumulate in organs such as the liver, muscle, heart, and pancreas, which is an essential pathophysiological abnormality of METS [5, 6]. Nonalcoholic fatty liver disease (NAFLD) is an example of ectopic fat accumulation in the liver. From simple steatosis, the disease may progress to nonalcoholic steatohepatitis (NASH) to hepatic cirrhosis and hepatic failure [7]. A number of studies suggest an association between NAFLD and METS [8–10]. The incidence rate of NAFLD is increased conspicuously in patients with DM concomitant obesity, while that ranges 40%-70% in DM patients [11] and 57%-98% in overweight and obese individuals [8]. Besides, a study [12] manifested an association between adipose infiltration of the liver and metabolic rate.

Few studies focused on the impact and clinical significance of ectopic fat accumulation in pancreas when compared with NAFLD in the past. But it has become the forefront of academic research recently [13]. The pancreas is a retroperitoneal organ that is hard for noninvasive investigations [14]. A high echogenicity of the pancreas is presented in routine transabdominal ultrasound examination. Advanced imaging technologies, such as computer tomography (CT), magnetic resonance imaging (MRI), and high-resolution proton magnetic resonance spectroscopy (1H-MRS), make it possible to evaluate and quantify pancreatic fat noninvasively and accurately [15, 16].

Pancreatic adipose infiltration is prevalent and is associated with at least a twofold increase in risks of type 2 diabetes mellitus (T2DM), METS, and hypertension [17, 18]. It is a risk factor for pancreatic cancer and precancerous pancreas as well [19, 20]. There seems to be some evidence to demonstrate that METS is related to pancreatic adipose infiltration [21, 22]. However, few investigators have drawn on any systematic research into the correlation between pancreatic adipose infiltration and METS [16]. Whether pancreatic adipose infiltration is caused by METS and obesity or a contributing factor to progression of METS would be a fruitful area for further work.

To sum up, we systematically reviewed and compared incidence of METS in adults with and without pancreatic adipose infiltration. We attempted to investigate correlation between pancreatic adipose infiltration and METS and to provide reference for clinical application of routine pancreatic adipose infiltration screening.

## 2. Methods

### 2.1. Literature Retrieval

This research was strictly followed Preferred Reporting Items for Systematic reviews and Meta-Analyses (PRISMA) statement [23]. PubMed, Embase, Cochrane Library, and Web of Science databases were searched to find relevant articles from inception to July 2021. Search items included “Pancreas,” “fatty,” “adipose,” and “Metabolic Syndrome,” etc. The specific strategy for literature retrieval was as follows: ((((Pancreas[MeSH Terms]) OR (Pancreas[Title/Abstract])) OR (pancreatic[Title/Abstract])) AND ((((fatty[Title/Abstract]) OR (adipose[Title/Abstract])) OR (steatosis[Title/Abstract])) OR (Fat[Title/Abstract]))) AND (((((((((Metabolic Syndrome∗[MeSH Terms]) OR (Metabolic Syndrome X[MeSH Terms])) OR (Metabolic X Syndrome[MeSH Terms])) OR (Insulin Resistance Syndrome X[MeSH Terms])) OR (Dysmetabolic Syndrome X[MeSH Terms])) OR (Reaven Syndrome X[MeSH Terms])) OR (Metabolic Cardiovascular Syndrome[MeSH Terms])) OR (Cardiometabolic Syndrome∗[MeSH Terms])) OR ((((((((Metabolic Syndrome∗[Title/Abstract]) OR (Metabolic Syndrome X[Title/Abstract])) OR (Metabolic X Syndrome[Title/Abstract])) OR (Insulin Resistance Syndrome X[Title/Abstract])) OR (Dysmetabolic Syndrome X[Title/Abstract])) OR (Reaven Syndrome X[Title/Abstract])) OR (Metabolic Cardiovascular Syndrome[Title/Abstract])) OR (Cardiometabolic Syndrome∗[Title/Abstract]))). Literature retrieval was completed independently by two investigators. Any discrepancies were resolved by a third investigator.

### 2.2. Study Selection

Study selection was completed independently by two investigators. Any discrepancies were resolved by a third investigator. Studies included met the following criteria: (1) diagnostic information about pancreatic adipose infiltration and METS and its components was provided; (2) a preliminary report on comparison of incidence rate of METS between adults with and without pancreatic adipose infiltration; (3) at least several results of METS, triglyceride (TG), fasting blood glucose (FBG), high-density lipoprotein (HDL), and hypertension (HTN) were reported; and (4) the study was a cross-sectional study, cohort study, or case-control study. Exclusion criteria were (1) duplicate publications, case series, case reports, reviews, conference abstracts, reviews, editorials, and letters and (2) lack of indicators required for this study or irrelevant data.

### 2.3. Data Extraction and Quality Assessment

Data extraction and quality assessment were completed independently by two investigators. Any discrepancies were resolved by the third investigator. Information that was isolated from literature included author information, publication year, country, study design, sample size. Patient features contained age, BMI, waist circumference, and incidence rate of pancreatic adipose infiltration. The primary endpoint was incidence rate of METS. Secondary endpoints were FBG, TG, HDL, and HTN.

The Newcastle-Ottawa Quality Assessment Scale (NOS) was used to generate a quality assessment of observational study. It consisted of selection (4 stars), comparability (2 stars), and outcome (3 stars). The total score was 9 stars. We found that a NOS score of 6 or more can be considered a good quality study. Any discrepancies between the two investigators were resolved by a majority opinion after all items involved were evaluated by the third investigator.

### 2.4. Statistics

Meta-analysis was completed by the Stata software 16.0. Consecutive data were presented as mean and standard deviation (SD). The specific efficacy was estimated by standardized mean difference (SMD) of consecutive outcomes and 95% confidence intervals (CIs). For binary outcomes, the combined estimation was the odds ratio (OR) and its 95% CI. The *I*^2^ statistic was used to assess heterogeneity of the included studies. Studies with *p* < 0.1 or *I*^2^ > 50% were considered to have significant heterogeneity, and therefore, a random-effects model was used. Otherwise, a fixed-effects model was initially employed in the analysis. Funnel plots were plotted to assess publication bias in outcome indicators.

## 3. Results

### 3.1. Literature Retrieval and Study Selection

A total of 1089 records were identified following the established retrieval strategy, and 435 duplicate records were excluded. Then, 634 reports were excluded by initial title and abstract screening, and 20 reports were reviewed in full text. Among them, 4 articles reported irrelevant data, and 5 articles lacked indicators required for this study. Finally, 11 studies were deemed eligible for inclusion [14, 22, 24–32]. Flow chart of study selection was plotted as Figure 1.

### 3.2. Study Characteristics and Quality Assessment

A total of 11 studies were deemed eligible for inclusion with 2,902 patients with pancreatic adipose infiltration and 14,225 participants without pancreatic adipose infiltration enrolled. 8 cross-sectional studies, 2 cohort studies, and 1 case control study were included. Characteristics and quality assessment of studies included are listed in Table 1. All of these studies were good quality studies with a NOS score of 6 or more.

### 3.3. Meta-analysis

#### 3.3.1. Incidence Rate of METS

9 studies were analyzed regarding the incidence rate of METS. The results presented a relatively high statistical heterogeneity (*I*^2^ = 73%, *p* < 0.01), and thus, a random-effects model was employed (Figure 2(a)). Taken together, there was a trend of increasing in incidence rate of METS (OR = 2.66, 95% CI: 1.89-3.75) of adults with pancreatic adipose infiltration when compared to those without the disease.

Sensitivity analysis was carried out to investigate potential sources of heterogeneity. Each item was assumed as a potential bias factor and source of heterogeneity. Then, sensitivity analysis was conducted, and forest plots were generated (Figure 2(b)). The results exhibited high heterogeneity.

#### 3.3.2. Secondary Endpoints

Some indicators are bound up with pancreatic adipose infiltration, including FBG, TG, HDL, and HTN.

8 studies compared FBG between patients with and without pancreatic adipose infiltration. The results presented a relatively high statistical heterogeneity (*I*^2^ = 89%, *p* < 0.01), and thus, a random-effects model was employed (Figure 3(a)). Each item was assumed as a potential bias factor and source of heterogeneity. Then, sensitivity analysis was conducted, and forest plots were generated (Figure 3(b)). The results exhibited high heterogeneity. Together, these results illustrated that there was a trend of increase in FBG (SMD = 0.54, 95% CI: 0.35-0.72) of adults with pancreatic adipose infiltration.

9 studies compared TG between patients with and without pancreatic adipose infiltration. The results presented a relatively high statistical heterogeneity (*I*^2^ = 84%, *p* < 0.01), and thus, a random-effects model was employed (Figure 4(a)). Each item was assumed as a potential bias factor and source of heterogeneity. Then, sensitivity analysis was conducted, and forest plots were generated (Figure 4(b)). The results exhibited high heterogeneity. Taken together, there was a trend of increase in TG (SMD = 0.39, 95% CI: 0.25-0.53) of adults with pancreatic adipose infiltration.

10 studies compared HDL between patients with and without pancreatic adipose infiltration. The results presented a relatively high statistical heterogeneity (*I*^2^ = 85%, *p* < 0.01), and thus, a random-effects model was employed (Figure 5(a)). Each item was assumed as a potential bias factor and source of heterogeneity. Then, sensitivity analysis was conducted, and forest plots were generated (Figure 5(b)). The results exhibited high heterogeneity. Together, these results displayed that there was a trend of decreasing in HDL (SMD = −0.29, 95% CI: -0.43~ -0.15) of adults with pancreatic adipose infiltration.

7 studies compared HTN between patients with and without pancreatic adipose infiltration. The results presented a relatively high statistical heterogeneity (*I*^2^ = 54%, *p* = 0.04), and thus, a random-effects model was employed (Figure 6(a)). Each item was assumed as a potential bias factor and source of heterogeneity. Then, sensitivity analysis was conducted, and forest plots were generated (Figure 6(b)). The results exhibited high heterogeneity. Taken together, there was a trend of increase in hypertension (OR = 1.68, 95% CI: 1.32-2.13) of adults with pancreatic adipose infiltration.

#### 3.3.3. Publication Bias

The funnel plots were basically symmetrical by visual observation, indicating no publication bias in the included studies (Figure 7).

## 4. Discussion

METS is featured as obesity, visceral fat accumulation, diabetes, hyperlipidemia, and hypertension [3, 4]. Pancreatic adipose infiltration is a component of METS similar to NAFLD. In the past, lack of appropriate survey tools that could enter the pancreas made it hard to assess pancreatic tissue in a timely and effective manner during laparoscopic or laparotomy [14]. Advanced noninvasive imaging technology makes it feasible to accurately detect and quantify pancreatic adipose [15, 16].

This study manifested by meta-analysis that incidence of pancreatic adipose infiltration was related to that of METS. Compared with adults without pancreatic adipose infiltration, adults with pancreatic adipose infiltration had an increasing trend of suffering from METS.

Some clinical features are bound up with METS [3], such as FBG, TG, HDL, and HTN. Meta-analysis investigated the association between them, and 11 studies were included with 17,127 participants enrolled. We found that levels of FBG (SMD = 0.54, 95% CI: 0.35-0.72), TG (SMD = 0.39, 95% CI: 0.25-0.53), and HTN (OR = 1.68, 95% CI: 1.32-2.13) were positively correlated with pancreatic adipose infiltration, while HDL level (SMD = −0.29, 95% CI: -0.43~ -0.15) was inversely correlated with pancreatic adipose infiltration.

Choi et al. [33] unveiled that pancreatic adipose infiltration was associated with systolic hypertension rather than diastolic hypertension. As such, our results displayed a significant trend of increasing in HTN (OR = 1.68, 95% CI: 1.32-2.13) in adults with pancreatic adipose infiltration. Ou et al. [34] illustrated that among independent risk factors such as obesity and cardiometabolic factors, pancreatic adipose infiltration may facilitate progression of diabetes. As detected by MRS or MRI, pancreatic fat content of subjects with T2DM is more than that of nondiabetic subjects [18, 35, 36]. Similarly, the proportion of T2DM patients in pancreatic adipose infiltration group was also higher than those in the nonpancreatic adipose infiltration group [26]. As such, we unraveled that FBG (SMD = 0.54, 95% CI: 0.35-0.72) in subjects with pancreatic adipose infiltration was higher than those with nonpancreatic adipose infiltration.

Our results based on 8 studies were consistent with a meta-analysis by Bi et al. [13] that pancreatic adipose infiltration was associated with METS and hypertension. We analyzed 11 studies with 34,074 participants enrolled. We also analyzed correlation between pancreatic adipose infiltration and FBG, TG, and HDL, which was not been dealt with previously.

The study was limited by high heterogeneity in the results of meta-analysis and failure in identifying possible bias factors and sources of heterogeneity. It is unfortunate that during literature retrieval, no randomized controlled trials were included regarding the comparison between adults with pancreatic adipose infiltration and those without the disease. Besides, one source of weakness in this study that could have led to regional and ethnic bias was that 9 out of 11 studies were in Asia.

To sum up, pancreatic adipose infiltration presented a correlation with METS, and it may be a phenotype of METS like fatty liver and a key to treating METS. These results indicated that routine pancreatic adipose infiltration screening had clinical significance. Nevertheless, the data used in this systematic review were mainly from studies in Asia. The pathogenesis of pancreatic adipose infiltration remains unclear. Hence, more clinical trials are warranted to unravel pathophysiology, long-term complications, clinical impacts, and the formulation of therapeutic regimens.

## Figures and Tables

**Figure 1:** Flow chart of study selection.

**Figure 2:** Forest plots of comparison in incidence rate of METS: (a) forest plot comparing the incidence rate of METS; (b) forest plot of prevalence of incidence rate of METS after sensitivity analysis.

**Figure 3:** Forest plots of comparison in FBG: (a) forest plot of FBG; (b) forest plot of FBG after sensitivity analysis.

**Figure 4:** Forest plots of comparison in TG: (a) forest plot of TG; (b) forest plot of TG after sensitivity analysis.

**Figure 5:** Forest plots of comparison in HDL: (a) forest plot of HDL; (b) forest plot of HDL after sensitivity analysis.

**Figure 6:** Forest plots of comparison in hypertension: (a) forest plot of hypertension; (b) forest plot of hypertension after sensitivity analysis.

**Figure 7:** Funnel plots: (a) METS; (b) FBG; (c) TG; (d) HDL.

**Table 1:** Baseline characteristics of studies included in the study.

Author	Year	Country	Sample size (*n*)		Gender (M/F)		Study design	Age, mean ± SD		BMI (kg/m^2^)		NOS
			Pancreatic adipose infiltration	Nonpancreatic adipose infiltration	Pancreatic adipose infiltration	Nonpancreatic adipose infiltration		Pancreatic adipose infiltration	Nonpancreatic adipose infiltration	Pancreatic adipose infiltration	Nonpancreatic adipose infiltration	
Lee	2009	South Korea	180	113	87/93	79/34	Cross-sectional study	45.4 ± 8.5	44.4 ± 9.7	26.5 ± 3.1	24.4 ± 3.2	6
Sepe	2011	USA	64	166	27/37	75/91	Cross-sectional study	62.6 ± 12.3	62.1 ± 14.1	29.4 ± 7.3	26.5 ± 6.3	6
Wu	2013	Taiwan	72	485	30/42	285/200	Case–control retrospective study	57.3 ± 12.4	20.7 ± 12.8	25.3 ± 2.7	23.7 ± 3.5	7
Wong	2014	Hong Kong	110	575	66/44	205/370	Cross-sectional study	52 ± 8	47 ± 11	24.7 ± 2.9	22.4 ± 3.5	7
Wang	2014	Taiwan	1297	6800	804/493	3672/3128	Cross-sectional study	56 ± 10	51 ± 11	25.8 ± 3.0	23.5 ± 3.0	6
Zhou	2016	China	365	825	223/142	367/458	Cross-sectional study	51.9 ± 13.1	47.7 ± 14.3	27.1 ± 3.2	24.4 ± 3.2	6
Wang	2018	China	53	1175	28/25	550/625	Cross-sectional study	57.7 ± 12.0	45.4 ± 14.2	25.8 ± 3.0	23.5 ± 3.0	7
Yamazaki	2018	Japan	214	106	192/22	82/24	Cohort study	53.8 ± 8.45	48.9 ± 8.8	24.45 ± 2.7	22.5 ± 2.5	6
Weng	2018	China	437	3895	271/166	1992/1903	Cross-sectional study	49.16 ± 8.12	47.91 ± 8.1	24.93 ± 2.83	23.12 ± 1.85	7
Milovanovic	2019	Serbia	84	59	55/29	42/17	Cross-sectional study	52 ± 13	52 ± 14	29.8 ± 4.1	28.5 ± 4.7	6
Chiyanika	2020	China	26	26	19/7	14/12	Cohort study	15.6 ± 1.3	15.7 ± 1.1	32.6 ± 3.4	32.1 ± 3.0	6

## Data Availability

The date and materials in the current study are available from the corresponding author on reasonable request.
